RETRACTED

# Clinical Brain Death with False Positive Radionuclide Cerebral Perfusion Scans

**DOI:** 10.1155/2015/630430

**Published:** 2015-06-08

**Authors:** Sindhaghatta Venkatram, Sara Bughio, Gilda Diaz-Fuentes

**Affiliations:** ^1^Division of Pulmonary and Critical Care Medicine, Bronx Lebanon Hospital Center, Bronx, NY 10457, USA; ^2^Albert Einstein College of Medicine, 1300 Morris Park Avenue, Bronx, NY 10461, USA; ^3^Department of Internal Medicine, Bronx Lebanon Hospital Center, Bronx, NY 10457, USA

## Abstract

Practice guidelines from the American Academy of Neurology for the determination of brain death in adults define brain death as “the irreversible loss of function of the brain, including the brainstem.” Neurological determination of brain death is primarily based on clinical examination; if clinical criteria are met, a definitive confirmatory test is indicated. The apnea test remains the gold standard for confirmation. In patients with factors that confound the clinical determination or when apnea tests cannot safely be performed, an ancillary test is required to confirm brain death. Confirmatory ancillary tests for brain death include (a) tests of electrical activity (electroencephalography (EEG) and somatosensory evoked potentials) and (b) radiologic examinations of blood flow (contrast angiography, transcranial Doppler ultrasound (TCD), and radionuclide methods). Of these, however, radionuclide studies are used most commonly. Here we present data from two patients with a false positive Radionuclide Cerebral Perfusion Scan (RCPS).

## 1. Introduction

The President's Commission report on “guidelines for the determination of death” culminated in proposing a legal definition that led to the Uniform Determination of Death Act (UDDA). The act reads as follows: “an individual who has sustained either (1) irreversible cessation of circulatory and respiratory functions, or (2) irreversible cessation of all functions of the entire brain, including brainstem, is dead [1].” Most state laws regarding brain death (BD) determination have their origin in the UDDA. In patients with clinical BD, a definitive test is mandated for confirmation. Apnea tests remain the gold standard for such determinations.

There are special circumstances where confirmatory ancillary tests are used, for example,

- uncertainty regarding the neurological exam (e.g., patients with unknown/unclear reason for brain death),
- patients with confounding factors, such as elevated levels of central nervous system sedatives or the presence of residual neuromuscular blockers,
- incomplete or unreliable neurological exam due to facial trauma or pupillary abnormalities,
- inability to perform an apnea test due to unstable respiratory or hemodynamic conditions (e.g., high oxygen or vasopressors requirements) [2].

RETRACTED

Confirmatory tests for BD include electrical activity tests (EEG and somatosensory evoked potentials) and radiologic blood flow examinations (contrast angiography, transcranial Doppler ultrasound (TCD), and radionuclide methods). EEG remains controversial due to the potential for artifacts and it is not widely accepted [3, 4]. Tests demonstrating the absence of cerebral blood flow remain commonly used. Of these, however, RCPS studies are the most common.

Here we report on two patients with false positive RCPS studies. This study was approved by the Institutional Review Board of Bronx Lebanon Hospital center.

## 2. Case Presentation

**Case 1 .**

A 71-year-old male presented with a sudden onset of slurred speech and bilateral leg weakness that resolved in 5 minutes. His medical history included hypertension, dyslipidemia, and previous stroke with no residual weakness.

Physical examination revealed normal vital signs and a NIH Stroke Scale International (NIHSS) score of 0 on neurological exam. Initial laboratory results were normal. The initial head CT scan showed no evidence of acute infarction. MRI results revealed small foci of acute infarction in the left posterior frontal and parietal vertex. Numerous remote cortical and subcortical basal ganglia and cerebellar infarcts were noted. The patient had ischemic white matter disease that was greater than expected for his age and a suspicious left vertebral occlusion. MR angiography of the head and neck showed intact intracranial circulation with patchy flow identified within the right vertebral artery, which appeared to be congenitally hypoplastic. We noted carotid stenosis with approximately 36% occlusion of the proximal right internal carotid artery (ICA) and 75% stenosis of the proximal left ICA. Transesophageal echocardiogram did not reveal any thrombi.

The patient underwent a left carotid endarterectomy; however, the postoperative course was complicated by acute stroke. He was liberated from the ventilator 4 days after the stroke. On day 6, he experienced cardiac arrest; he was resuscitated with return of spontaneous circulation (ROSC) in 20 minutes. Subsequently, he had two more episodes of cardiac arrest and was successfully resuscitated with ROSC in 8 and 5 minutes, respectively. He developed shock and multiorgan failure. His neurological status deteriorated with a GCS of 3 and the absence of brainstem function, except for a few trigger efforts. He remained hemodynamically stable with an unchanged neurological exam. Brain perfusion imaging was performed at his family's request and showed results consistent with BD (Figure 1). He continued to have spontaneous breathing after the cerebral perfusion study, and no other ancillary tests were performed. His family requested palliative care and he was transferred to a hospice, where he died from cardiac arrest.

RETRACTED

**Case 2 .**

A 46-year-old male was admitted to our hospital after his wife found him on the floor in a pool of vomitus with bladder and bowel incontinence after a witnessed seizure.

His medical history included hypertension, dyslipidemia, diabetes mellitus type II, chronic kidney disease, and history of stroke without residual weakness.

Physical examination revealed an obese patient with tachycardia (heart rate, 107), accelerated hypertension (blood pressure, 189/102), and tachypnea (respiratory rate, 36). He had agonal breathing, was gazing to the left, and could move his left arm but not his right arm. His gag reflex was present. His pupils were equal and reacted to light. His GCS scale was 3/15. Cardiovascular, respiratory, and abdominal examinations were unremarkable. He required intubation for airway protection. A head CT scan revealed a large acute intraparenchymal hematoma with a midline shift from the left to right and a potential uncal herniation. He underwent emergent left-sided craniotomy to evacuate the hematoma. The GCS scale improved to 6 (E1V1M4) on the third day after surgery. His hospital course was complicated due to failure to wean, persistent fever, nosocomial pneumonia, and urinary tract infections. His neurological status did not improve, and he underwent tracheotomy and was transferred to a regular ward. The patient received lorazepam (2 mg) for agitation on his first day in the ward. On the second day during rounds, the clinical exam revealed normal pulse and blood pressure, no spontaneous breathing, GCS of 3, and the absence of brainstem function. The patient was suspected to be clinically brain dead. However, an apnea test could not be performed in the ward. Therefore, a cerebral perfusion scan was performed 24 hours later, with results consistent with brain death. His family was informed of the findings and mechanical ventilation was continued to allow the family time to gather. On day 3 in the ward, the patient was noted to have spontaneous eye opening with a change in neurological status. Due to the new clinical developments, a repeat perfusion scan was done 48 hours after the first scan. This second scan again revealed no cerebral perfusion (Figures 2 and 3). No other ancillary tests were performed. The patient was transferred to a hospice and died a week later.

## 3. Discussion

Brain death can be determined by a skillful neurological exam and confirmed by an apnea test. In situations where components of the clinical exam are unreliable or apnea tests cannot be performed, confirmatory ancillary tests are required. Commonly used ancillary tests in adults include EEG, cerebral angiography, nuclear scan, TCD, CT angiography (CTA), and MRI/MRA. The preferred tests at most institutions are nuclear scans or cerebral angiography. Of the many attributes of an ideal ancillary test, the most important is a lack of false positives.

RETRACTED

RCPS was performed in both of our patients. Most confirmatory studies for BD, including RCPS, can be associated with false positives and false negatives. A false positive nuclear scan occurs when the nuclear scan reveals no perfusion and confirms BD, but the clinical exam is not consistent with BD [5–7]. False negative scans reveal perfusion when there is no clinical evidence of brain function by clinical exam. In a review of 229 procedures done in 219 patients, the sensitivity of radionuclide angiography was 98.5%; five cases were not BD but had no flow [8]. In 2010, Joffe et al. presented a pediatric case similar to ours and reviewed the literature on cerebral perfusion scans [9]. In this review, the sensitivity of the perfusion scan was 77.8%; however, their study was confounded by the lack of complete clinical data.

The presence of blood flow in radionuclide angiography in patients with clinical BD has been previously explained in detail [10]. This includes differences in the sensitivity of both clinical exam and blood flow, ancillary tests performed relatively soon after the neurologic event, technical problems evaluating brainstem perfusion, and differences between blood flow and function as indicators of irreversible loss of brain function.

Preserved brainstem function in the absence of blood flow is scarcely reported. However, this likely reflects an inherent bias because ancillary tests are seldom ordered in patients with preserved brainstem function. A lack of blood flow in patients without clinical evidence of BD can be explained only when anterior views are used. Spieth et al. reported the importance of lateral projection in reporting BD because lateral views view cerebellar blood flow in patients without clinical evidence of BD can be explained only when anterior views are used [11]. Another cause of the lack of blood flow is the use of central nervous system (CNS) depressants that mask the clinical exam; however, blood flow studies are rarely performed in these situations. In our study, blood flow was examined in the first patient due to disparities in the neurological exam. The second patient had clinical evidence of BD that was confirmed by lack of blood flow. He regained brainstem function, but a repeat blood flow analysis also showed a lack of blood flow, which was confirmed by two radiologists. It is very unlikely that lorazepam (2 mg) resulted in CNS depression, thereby mimicking brain death 24 hours after administration.

RETRACTED

A review of all radionuclide scans performed at our institution for clinical BD from April 2010 to May 2014 revealed 21 studies performed on 20 patients, including the patients presented in this study (Table 1). The indication for all of these studies was the inability to perform apnea tests. In one patient with clinical evidence of brainstem function, a perfusion scan was done per the request of the patient's family. Of the 19 studies performed in clinically brain dead patients, 18 confirmed BD patients (true positives) either were removed from ventilator support or had organs donated. In one patient, the cerebral perfusion scan was a false negative, because the patient showed subsequent brainstem activity. A repeat scan in the same patient with continued brainstem activity showed no perfusion, thus indicating a false positive. A perfusion scan done in one patient with brainstem function revealed no cerebral blood flow (CBF), also indicating a false positive. The sensitivity of cerebral perfusion scans in our series was 94.74% (95% CI, 73.9–99.12) with a positive predictive value of 90%. There were no true negatives, because both patients with brainstem function did not have flow; thus, there was a specificity of 0% (95% CI, 0–80.7%). However, specificity analyses should be interpreted with caution because RCPS scans are not routinely performed on patients with brainstem activity.

In our series, two patients with brainstem activity had RCPS results consistent with brain death. The common factor in both patients was surgery. In the first patient, carotid endarterectomy was performed, which was followed by a subsequent stroke. The second patient underwent craniotomy for intracranial bleeding. We believe it is very unlikely that there is any association between head surgery and false positive scans.

The agents used in cerebral perfusion studies include TC-99m pertechnetate, TC-99m glucoheptonate, TC-99m DTPA, and TC-99m HMPAO. Of these agents, TC-99m pertechnetate, TC-99m glucoheptonate, and TC 99m DTPA (TC) do not cross the blood brain barrier. TC-99m HMPAO is lipophilic and can cross the intact blood brain barrier and localize in gray matter proportional to perfusion for delayed imaging. A study comparing these agents showed that TC-99m HMPAO is superior for cerebral perfusion studies in order to determine BD [12, 13]. At our institution, nuclear scans are routinely performed with TC 99m DTPA (TC) and immediate anteroposterior (AP) and lateral views are acquired. After 20 minutes, delayed views are acquired.

RETRACTED

In our patients, an absence of flow was observed in all views. It is possible that some blood flow to the brainstem that was not detected by radionuclide scan accounted for the disparity.

There was no neurological recovery in our patients, who both eventually died during palliative care.

## 4. Conclusion

Our report confirms that radionuclide scans are less than ideal ancillary tests because rare false positives have been observed. Because there are significant implications for discussions with families regarding patient care and the potential for organ donation, physicians involved in this end of life event should be aware of the potential pitfalls of ancillary tests used for BD determination.

## Figures and Tables

**Figure 1:** Patient #1. RCPS showing anterioposterior and lateral immediate and delayed images revealing no cerebral blood flow (empty skull sign).

**Figure 2:** Patient #2. RCPS showing anterior and posterior views with no cerebral blood flow.

**Figure 3:** Patient #2. RCPS summative view.

**Table 1:** Summary of 21 radionuclide scans for brain death determination at our institution.

	No uptake	Uptake	Comments
Clinically BD	18	1	One patient initially declared clinically BD showed spontaneous eye opening

Clinically not BD	2	0	

## Abbreviations

BD: Brain death
RCPS: Radionuclide Cerebral Perfusion Scans
UDDA: Uniform Determination of Death Act
EEG: Electroencephalography
TCD: Transcranial Doppler ultrasound
CVA: Cerebrovascular accident
CT: Computed tomography
GCS: Glasgow Coma Scale/Score
CTA: CT angiography
MRI/MRA: Magnetic resonance imaging/magnetic resonance angiogram
CNS: Central nervous system
CBF: Cerebral blood flow
TC: Technetium.
